The article "Cross-Disciplinary Application for Qualitative Magnesium Corrosion Assays" was published in 2022. Journal: Bioinorg Chem Appl.

# Cross-Disciplinary Application for Qualitative Magnesium Corrosion Assays

**DOI:** 10.1155/2022/8289447

**Published:** 2022-06-28

**Authors:** Xinzhe Gao, Yunhan Sun, Qi Jia, Eui-Seok Lee, Heng Bo Jiang

**Affiliations:** ^1^The Conversationalist Club, School of Stomatology, Shandong First Medical University and Shandong Academy of Medical Sciences, Tai'an, Shandong 271016, China; ^2^Department of Oral and Maxillofacial Surgery, Graduate School of Clinical Dentistry, Korea University, Seoul 08308, Republic of Korea

## Abstract

At the moment, unserviceable magnesium implants make a good case in point for further responsible study in this field. Whether we are willing to admit it or not, existing methods for corrosion monitoring are exposed to susceptibility and instability. Interdisciplinary theories and the existing corrosion experiments were combined based on their various merits for developing an accurate and precise corroding experiment for Mg/Mg alloys. We used the water-soluble tetrazolium-8 (WST-8) reagent to further complete the immersion experiment. The color change of the solution reflects the rationale of corrosion, followed by monitoring the degree of corrosion. The feasibility of this idea will be demonstrated.

## 1. Introduction

Magnesium, as a fundamental kind of dietary trace element, can be controlled by homeostatic mechanisms in organisms [1]. Considering the merits of magnesium and magnesium alloys, its application in clinical implants seems like a sure choice [2–4]. Yet, studies have shown that there is still a major problem with the biodegrading behavior of magnesium/magnesium alloys that remains to be solved [5, 6]. Data from existing studies have shown that under the conditions to which the metallic implants are exposed to, both the rapid degrading process and intricate corroding mechanism are adversely affected [7, 8]. Regarding the complex corroding mechanism of Mg/Mg alloys, it is thought to simply be an electron-transfer model where the Mg in the alloy loses electrons to generate Mg^2+^ (also called the anodic dissolution) [9]. The correct measurement of corrosion rate and the affecting parameters are imperative when implementing corrosion control. Surveys, for instance, such as the one conducted by Nicholas Travis Kirkland and Nick Birbilis, [10] have analyzed and sorted past commonly used experiments. In addition, the study enumerated most of the instructive techniques.  Table 1 compiled the advantages and disadvantages of common methods.

From the perspective of perfecting and compensating for the drawbacks of traditional methods, researchers paid significant effort to this endeavor even when there is no perfect way to characterize the corrosion rate or behavior of Mg/Mg alloys in Hank's balanced salt solution (HBSS) immersion. Hank's balanced salt solution (HBSS) has a chemical composition similar to that of human blood plasma, which is a suitable electrolyte that simulates the body fluid environment for immersion experiments. It is worth mentioning that Shanmugam et al. [18] tried from an advantageous motivation to optimize and improve the immersion experiment. However, given that the reagent was susceptible to change in pH, the experiment only reflected the corrosion process indirectly. At the same time, the hydrogen bubbles in the reaction process on the solution acidity and alkalinity [19, 20]. The environmental conditions are mainly determined by the corrosion solution used, [9] which means that the solution composition needs to change to a great extent without affecting the corrosion process. This experiment serves as a reminder that if the reagent is not ideal, it is susceptible to the influence of the environment, the product, and the detection time [21]. In light of this, we are dedicated to finding more stable indicators reflecting the corrosion rate so that the results could better directly evaluate the resistance of the magnesium substrate than other studies.

The article "Cross-Disciplinary Application for Qualitative Magnesium Corrosion Assays" was published in 2022. Journal: Bioinorg Chem Appl.

In biochemical experiments, the measurement of live cell counts often requires more stable and sensitive methods and reagents [22, 23]. The reagent water-soluble tetrazolium-8 (WST-8) can be used in quantitative experiments in this field, which gives it the potential to become an indicator for monitoring the degree of corrosion [24]. When corrosion occurs due to the loss of electrons, WST-8 as a reactant is reduced from the tetrazolium salt to the formazan product by Magnesium. Formazan is a strong orange substance that can be detected in the absorbance range between 430 and 550 nm [25–27].

This investigation aims at exploring the correlation between the optical density (OD) of HBSS, modified with the addition of WST-8 kit, and immersion time as a more accurate option for monitoring the degradation rate of Mg/Mg alloys [28]. The experimental work presented here provides a method to evaluate Mg/Mg alloys with diverse nuances, or to rank the specific type of surface finished material prepared with a small variation in the processing period, in terms of different degrees of corrosion.

However, although *in vivo* testing is certainly intuitive for a final result, the extensive usage of experimental animals is unrealistic and unethical. Thus, HBSS is used to mimic an ideal situation for all immersion experiments [29, 30]. Therefore, in this study, the *in vitro* tests are chosen to draw reasonable conclusions.

The article "Cross-Disciplinary Application for Qualitative Magnesium Corrosion Assays" was published in 2022. Journal: Bioinorg Chem Appl.

## 2. Materials and Method

### 2.1. Test Specimens

Three representative magnesium alloys were investigated in this study, that is, AZ31, AZ41, and AZ91 (Dongguan, China). The sheet was laser-cut into types of disc (10 mm × 9 mm × 7 mm). The composition of these alloys is listed in Table 2. The chemical composition of the alloy was evaluated by wavelength-dispersive X-ray fluorescence (WDXRF) before processing. The metal content of the WDXRF spectral data was evaluated by a nonstandard method. The results showed no significant differences between the samples [21, 31].

All the samples were cast into a cube shape following a standard procedure. Prior to all experiments, the specimens were ground and polished with ^#^2000 SiC paper in pure ethanol. Then, the polished samples were ultrasonically cleaned for 10 minutes in both distilled water and ethanol and dried by a compressed air gun. We then divided the test specimens into different experimental groups where each group contained samples with different compositions but the same dimensions. Every sample was discarded after being tested. Additionally, a blank control group was needed for the *f*-test.

### 2.2. Immersion Test

The immersion study is a well-established approach in corrosion investigation similar to the commonly used mass loss (ML) test. The ML test is widely used in the corrosion resistance study of magnesium alloys, which has the advantage of good accuracy and operability. The mass deficiency of the sample after redox reaction in a specific solution environment for a certain time is recorded to evaluate the corrosion rate. The assay process takes place in a specific liquid environment and is therefore also considered an immersion experiment. This long-term experiment is widely available and has been used in numerous studies [32, 33]. The chemical compositions of electrolyte HBSS are listed in Table 3. The testing solution was sterilized by filtration through a 0.22-*μ*m membrane filter and poured into sterile glass bottles. Prior to testing, the bottles with HBSS were sealed and kept under isothermal condition at 37°C overnight. The ratio of the HBSS volume on the sample area was 20 ml·cm^−2^. Afterward, one experimental group was aseptically immersed in each bottle with fluid. Then, all bottles were placed in an air incubator for one week under static environmental conditions. According to the Standard ASTM G1-03, the product-removal process was used after the immersion period to determine the state of the corrosion. All tested specimens were ultrasonically cleaned in a 20% chromium trioxide solution for 1 min, rinsed with pure ethanol, and dried. The percentage of ML testing was calculated as followed.

The article "Cross-Disciplinary Application for Qualitative Magnesium Corrosion Assays" was published in 2022. Journal: Bioinorg Chem Appl.

All kinds of samples, AZ31, AZ41, and AZ91, were treated and immersed in HBSS for 1800 minutes. The samples were taken out and washed with chromic acid to remove the insoluble salt layer formed on the surface. The samples were then air-dried. The remaining mass was measured to determine the mass loss by equations (1) and (2). From these equations, the mass loss rate of magnesium alloys is calculated as follows:

(1) $$\begin{array}{c} M_{\text{loss}}=M_{\text{0}}-M_{\text{retai}}, \end{array}$$

(2) $$\begin{array}{c} {\text{Mass}}_{\text{Loss}}\left(\%\right)=M_{\text{loss}}÷M_{\text{0}}, \end{array}$$

The remaining mass is represented by *M*_loss_, the original mass of the magnesium alloy is represented by *M*_0_, and the mass loss is represented by *M*_retain_.

### 2.3. Electrochemical Tests

The corrosion tests were performed at laboratory temperature under aerated conditions. During the immersion test, other two experimental groups were electrochemical-tested separately. The electrochemical tests were conducted with a stabilizer (VersaSTAT 3 : 300, AMETEK, US). The corrosion cell, where the tests will be carried out, was a 3-electrode set-up. Pure graphite was applied as the counter electrode, Ag/AgCl/Sat-KCl as the reference electrode, and the alloys of the experimental group as a working electrode. A single-tube capillary tube was placed next to the sample to reduce the IR drop between the reference electrode and the working electrode. 1 L of commercial HBSS (WELGENE Inc., Korea) was used, and the temperature of the electrolyte was maintained at 37°C by using a circulating water heater.

The electrochemical impedance was measured at a frequency between 100,000 and 0.1 Hz with an amplitude voltage of 5 mV on the *E*_corr_. During the performance of the impedance measurements, requirements for linearity and casualty were met. At a relatively low perturbation, controlling the response of the perturbation within the linear range was not a problem. To achieve the casualty of measurements, all responses should be caused by the perturbation rather than other environmental variables. To evaluate the corrosion resistance, 0.1 Hz was selected as the minor frequency and 20 minutes was chosen as the time limit. The extended period was adopted to help understand irreversible corrosion at relatively rapid and short periods.

After EIS measurement, the potentiodynamic polarization (PDP) tests for experimental group 3 were carried out to determine the polarization resistance value as an evaluation of corrosion resistance. The PDP tests mirror the relationship between the corrosion current density and the corrosion potential of the sample in a short time. Theoretically, the detection cathode produces a product layer. However, the whole process has a fast scan rate and magnesium alloys are a chemically diverse and active sample to detect. Therefore, the effect of this procedure on the results might be irrelevant. This is an electrochemical test method widely used for corrosion resistance studies of magnesium alloys. To better understand the rapid corrosion resistance of these alloys, the specimens were polarized in the electrolyte (HBSS) from −1.9 V to −0.5 V, using a scan rate of 1 mV/s, to determine the polarization resistance value [21].

The article "Cross-Disciplinary Application for Qualitative Magnesium Corrosion Assays" was published in 2022. Journal: Bioinorg Chem Appl.

### 2.4. Formazan Check Test (*f*-Test)

Changes in the concentration of the WST-8/formazan in the solution cause a change in the color. Due to the formation of the product generated by the oxidized WST-8, a group of experimental samples could be measured by the *f*-test. The WST-8 kit, containing 5 mM WST-8 and 0.2 mM 1-MPMS, was obtained from Sigma-Aldrich (St. Louis, Missouri, USA). The reaction conditions, including the buffer solution, substrate alloys, and the concentration of WST-8, were optimized for determining corrosion behavior. In an attempt to retain the characteristics of the simulated body fluid and produce natural conditions for magnesium alloy corrosion, the employed HBSS was sterilized and kept under isothermal conditions at 37°C overnight. The sample preparation process as well as the solution preparation process included a complete sterilization and disinfection step. The lowest possible level of microorganisms is guaranteed.

To obtain the actual color changes of the reagent, the WST-8 was diluted with treated HBSS solution before the assays. The WST-8 supplied by the kit was mixed with the treated HBSS at a ratio of 1 : 10. Then, the *f*-test reagent (HBSS blended with WST-8) was poured into different test tubes and the different samples were monitored separately. The total volume of the *f*-test reagent in the different test tubes was determined according to the superficial area of the Mg alloys. As shown in Figure 1, the WST-8 collects the electrons released by the oxidation of magnesium, which can be tested through the formazan reagent.

Further details include adjusting the system by 1 mL for each square centimeter. In order to avoid assay interference, the blank reaction was carried out in the absence of magnesium alloys. After monitoring the change in the OD value of the blank group after a certain time, it was found that this figure did not show noticeable changes. The changes of the reagents themselves could be neglected, so that the values of the blank group in Figure 2 may serve as a control during the experimental phase. The microplate reader was used to determine the OD value at 450 nm of the reagent in the tubes. Prior to this observation, the centrifugation and filtration procedures of the solution were omitted. The supernatant from the reaction of the static experimental group was compared with the filtered solution after centrifugation. The effect of both treatments on the OD value was found to be negligible. Meanwhile, this experiment aims at establishing an evaluation system for real-time monitoring of the corrosion degree of magnesium alloy. From these two starting points, the centrifugation and filtration procedures were considered to be skipped. The immersion time was set at a total of 1800 min (30 h), while the results were obtained at specific intervals of 20 min, 60 min, 120 min, 240 min, 480 min, and 1800 min.

The article "Cross-Disciplinary Application for Qualitative Magnesium Corrosion Assays" was published in 2022. Journal: Bioinorg Chem Appl.

### 2.5. Feasibility Analysis of the *f*-Test

The mass loss tests were carried out during the Mg alloy immersion period. Changes in mass were recorded after one week, which was used to determine the degree of corrosion. At the same time, 100 *μ*L of testing reagent was sampled for spectrophotometric analysis, conducted by the microplate reader, and the OD value at 450 nm was determined. The OD at 450 nm was recorded in the absence of substrate alloys for background subtraction. After each sampling, 100 *μ*L of HBSS was added in order to complement the initial reagent volume.

Three groups of samples, AZ31, AZ41, and AZ91, were soaked in Hank's solution with WST-8, and the OD value at 450 nm was measured at various intervals, while the Mg^2+^ concentration was measured using 100 *μ*L solution and calculated according to equation (3). According to the absorbance and Mg^2+^ concentration data, a plot of OD-Mg^2+^ yields a concentration curve:

(3) $$\begin{array}{c} C_{\text{Mg}}^{2+}=M_{\text{loss}}÷V_{0}, \end{array}$$

where *M*_loss_ is the mass loss of the experimental material and *V*_0_ is the initial volume of the HBSS solution.

## 3. Results and Discussion

### 3.1. Mass Loss (ML) Experiments

As seen in Figure 3, AZ41 reported significantly lower corrosion resistance than the other two samples. Moreover, there was no noncorrosive shedding of any sample. Through this long-term experiment, the percentage of mass loss after one-week immersion was 0.10%, 0.22%, and 0.52% for AZ91, AZ31, and AZ41, respectively. Since no chromic acid-soluble precipitate is formed, the percentage can be directly calculated, as shown in Table 4. Thus, the conclusion can be drawn that the order of highest corrosion resistance of these three tested alloys was AZ91 > AZ31 > AZ41.

In general, the results obtained from ML tests are accurate and dependable [9]. It is assumed that the corrosion layer removal problem is minimized as corrosion is relatively easy to observe. ML experiments require a relatively wide range of degrees of corrosion to accurately measure mass changes. In addition, although ML experiments reveal the physical quantities of corrosion that have occurred, they do not leak into the mechanisms involved in the corrosion process [39].

The article "Cross-Disciplinary Application for Qualitative Magnesium Corrosion Assays" was published in 2022. Journal: Bioinorg Chem Appl.

### 3.2. Potentiodynamic Polarization (PDP) Experimental Analysis

The corrosion parameters of the three tested specimens were determined by dynamic polarization experiments, as shown in Figure 4. From Figure 4, it can be seen that the corrosion resistance can be ranked from the highest to the lowest as AZ91 > AZ41 > AZ31. From the PDP curves above, it can be seen that the green curve (AZ91) shows the lowest current density of 2.0 × 10^−4^ A/cm^2^. Since the polarization resistance (Rp) is inversely proportional to the corrosion current density, the corresponding polarization resistance is the largest, indicating that the sample (the green curve, AZ91) has better corrosion resistance [40]. The current density (*i*_corr_) measured for the AZ41 and AZ31 (represented by the red and black curves respectively) is very similar. Therefore, the corrosion voltage (*E*_corr_) in the data was used to differentiate the corrosion resistance of the two. By comparing the corrosion tendencies of both under the same conditions, it was found that the corrosion voltages of samples AZ41 and AZ31 were −1.27 V and −1.29 V, respectively. It can be concluded that samples AZ41 have better corrosion resistance during the electrochemical experiments. It should be noted that the PDP experiment indicates the severity of corrosion at a selected point in time (in the form of a current densitometer) and that the corrosion rate in terms of current density and corrosion voltage is considered to be accurate.

### 3.3. Corrosion Impedance Capability Analysis

The results show that there are clear capacitive reactance arcs. The capacitive reactance arcs in the high-frequency region indicate that the electrode reaction corresponding to alloy corrosion is controlled by electrochemical reactions, that is, electron transfer. The resulting radius in the middle- and low-frequency regions is related to the corrosion resistance of the alloy. The Nyquist plots demonstrate that the larger the radius, the lesser it is possible to transfer electrons at the microlevel [41]. This also shows that the AZ91 alloy has high corrosion resistance, the best corrosion resistance among the three tested alloys. Because the experimental data in the low-frequency region have crucial significance for determining the impedance of the tested alloys, we determined their impedance values and ranked the samples in the following order: AZ91 > AZ41 > AZ31. In Figure 5(b), the frequency values decreased gradually from 100 kHz to 0.1 Hz. At about 7 Hz, the electrochemical impedance differences of the three alloys were clearly distinguishable, followed by a gradual increase. Hence, the impedance sequence is AZ91 > AZ41 > AZ31. These results are consistent with that of the dynamic polarization curve.

The article "Cross-Disciplinary Application for Qualitative Magnesium Corrosion Assays" was published in 2022. Journal: Bioinorg Chem Appl.

Moreover, the EIS tests provide near-instant information about the surface impedance, as affected by small polarization. This impedance is inversely proportional to the corrosion rate and can be used as an indicator of dissolution.

It is worth mentioning that there are differences between the results of the two experimental systems [42]. After demonstrating the electrochemical experiment results (experiment with EIS in Figure 5), the electrochemical and ML immersion experimental results were compared. Based on ensuring accuracy for the two experiments, we found subtle differences in the experimental results on whether AZ31 or AZ41 presented better corrosion resistance. In general, the results obtained from ML tests are accurate and dependable. It is assumed that the corrosion layer removal problem is minimized and that the corrosion is relatively obvious. ML experiments require a relatively wide range of degrees of corrosion to accurately measure mass changes. In addition, although ML experiments involve the physical quantities of the corrosion that occurred, this approach does not leak into the mechanisms involved in the corrosion process. However, the polarization curves showed that the alloys exhibited different corrosion potentials and phases for anode and cathode reaction kinetics (Figure 4). This behavior is particularly important for more physiologically realistic media because organic components, such as amino acids and proteins, have different effects on different parts of the reaction. The two experimental systems, which should be complementary, resulted in different conclusions. By analyzing both systems, they are generally considered to be accurate. However, there is a slight difference between the two systems in determining the corrosion resistance of an alloy. The differences between the samples were negligible, and the problem may arise from the time dimension of the analysis. This perception was also mentioned in the study of Chen et al. [43]. Thus, in consideration of the short electrochemical test time and the long immersion time, the change process and time point of two alloys with similar corrosion resistance, AZ31 and AZ41, were missed when observing the results.

The article "Cross-Disciplinary Application for Qualitative Magnesium Corrosion Assays" was published in 2022. Journal: Bioinorg Chem Appl.

### 3.4. Formazan Check Test (*f*-Test)

The OD values of each experimental group at 20 min, 60 min, 120 min, 240 min, 480 min, and 1800 min were recorded, and the results are plotted in Figure 6. It is worth mentioning that there were two pivotal points in the line chart of Figure 6, which are 240 min and 480 min.

At 240 min, there was a change in gradient and this pivotal point divides the graph into two different tendencies. At about 230 min, the degree of corrosion of the three alloys changed. At the beginning of the experiments, within the first approximately 230 minutes, the amount of corrosion was AZ31 > AZ41 > AZ91. During the initial stage of the WST-8 optimized immersion experiment, AZ31, represented by black dots, had a high degree of corrosion compared to the other tested samples, which is reflected in Figure 6 by the relatively high OD value. Moreover, it also indicates that AZ41 has better corrosion resistance than AZ31 after a short time interval, which is also reflected in electrochemical tests. However, at 240 min, AZ41 began to corrode more than AZ31 meaning that in the later stages of the experiment, AZ31 showed stronger corrosion resistance, which was consistent with the results of the mass loss tests.

Secondly, the significant differences in corrosion resistance for the tested alloys are shown at around 480 min. These results may have implications for the application of the two alloys.

By monitoring the blank control group (the blue line) for over 1800 min, it can be used to detect systematic interference by other unpredictable factors. When WST-8 is reduced to form the formazan product, it was found that other factors had no significant influence and that the color change of the solution could be attributed to the formazan product [44]. Moreover, the reaction was only related to the gain and loss of electrons associated with the REDOX reaction. The pH value, among other factors, did not affect the preparation of formazan by WST-8 [45]. During the monitoring of the *f*-test, the solution appeared to have a different color than in previous biochemical experiments (Figure 4). We speculate that the reason for this is the appearance of a macroscopically visible change in the mass of the magnesium alloy sample caused by corrosion. The electrons transferred in this change are much larger than colorimetric dehydrogenase detection for cell viability [24].

### 3.5. Feasibility Analysis

Based on the understanding above, we determined the characteristics of several experiments and analyzed the formazan check test (*f*-test). During HBSS immersion with WST-8, this approach can also be used for mass loss detection of naturally corroded alloys using the characteristics of the simulated body fluids. Due to the oxidation of magnesium during the corrosion process, magnesium loses electrons and forms magnesium ions in solution. At the same time, this process leads to two results for the HBSS experiment system optimized by WST-8. First, mass defects happen due to corrosive dissolution. Then, the electron loss of the magnesium alloy results in a reduction reaction of WST-8 to generate the heavy stained formazan product. That is to say, a single corrosion manifests as two different results. Therefore, in Figure 7 we compared the intercorrelations between these two results to see whether the experimental results are in direct proportion. According to the graph, the accuracy and feasibility of the *f*-test can be determined, which is the degree of corrosion of the magnesium alloy as reflected by the OD value.

The article "Cross-Disciplinary Application for Qualitative Magnesium Corrosion Assays" was published in 2022. Journal: Bioinorg Chem Appl.

We randomly selected 3 time points from the 3 tested groups containing alloy samples. The value of dissolved alloys, which is the concentration of magnesium ions in solution, was approximately calculated. The results were analyzed and found to be directly proportional. The most noteworthy point is that the WST-8 reagent is highly sensitive to the captured electrons, [46] as reported by numerous previous studies. This also reflects its accuracy in monitoring the degree of corrosion from the nature of the corrosion environment.

## 4. Conclusion

Based on the results above, the following conclusions can be drawn:

1. The results suggest that the formazan check method (*f*-test) is a sensitive and rapid method for determining the corrosion behavior of magnesium and magnesium alloys that can be further applied for the high-accuracy screening and selection of Mg/Mg alloys.
2. According to the principle of charge transfer, which is the essence of alloy corrosion, a novel method can be proposed to comprehensively and accurately determine the degree of corrosion of magnesium alloys. This is of great significance and experimental prospect for further research in this field.
3. As a corrosion monitoring experiment, the *f*-test, optimized by WST, has shown good performance in terms of accuracy, efficiency, and reproducibility. At the same time, this interdisciplinary direction also serves as an important reminder for further research and application in the field of alloy corrosion.

## Figures and Tables

**Figure 1:** Symbolic representation of the main chemical reaction with the visible reagent color changes during the *f*-test [34–38].

**Figure 2:** Color of the control and experimental groups in the *f*-test. As corrosion continues to occur, the color of the experimental group gradually changes: light salmon (OD = 0.05), olive (OD = 1.10), olive drab (OD = 1.80).

The article "Cross-Disciplinary Application for Qualitative Magnesium Corrosion Assays" was published in 2022. Journal: Bioinorg Chem Appl.

**Figure 3:** The weight change of the tested specimens after a one-week immersion experiment (the red, green, and black bars represent three alloys, respectively).

**Figure 4:** The corrosion resistance of the specimens by polarized dynamic potential experiment.

**Figure 5:** The corrosion impedance capability of each alloy in EIS experiments. (a) The arc radius dimensions symbolizing the corrosion impedance properties of the tested alloys. (b) Directive variation curve of impedance with frequency (Hz).

**Figure 6:** The OD values of the solutions monitored with a microplate reader along with the immersion time.

**Figure 7:** The results of the feasibility analysis of OD value and concentration of magnesium ions dissolved in the HBSS solution. The concentration of magnesium ion was taken as the *X* value, and the OD value of the solution monitored at the time point was plotted as the *Y*.

**Table 1:** Summary of available techniques.

Method	Advantages	Disadvantages
Mass loss experiment	Low cost [11]	Removing corrosion products from the surface may result in inaccuracies [12]
	An exposed surface can be provided to assess corrosion surface morphology [12]	It is dangerous to use chromic acid solution to clean corrosion products
	Easy set-up and performance	Only an average corrosion rate is provided, and it usually varies over time [6]
	Easy to control environment	Provides no information on corrosion mechanisms [11, 12]
		The ratio of surface area to medium needs to be precisely controlled, and pH is proportional to it [11]

Hydrogen evolution measurement	Low cost [11]	H_2_ bubbles are usually attached to the wall of the tube, leading to an
	The results were not affected by corrosion products	Underestimate of the rate of HE [11]
	Real-time measurement [13]	Not suitable for corrosion-resistant metals and short time experiments [11]
	Hydrogen is produced in the human body, H_2_ measurement is vital [14]	Dissolution of H_2_ in solution affects the results [15]

pH meter	Low cost [11]	Metal hydrolysis may also affect the pH of the solution
	Accurate detection in real time	Real-time measurement is limited by the time required for titration, which limits the evaluation of cathodic kinetics [12]
	Easy set-up and maintain	In vitro experiments should try to avoid pH changes [11]

Potentiodynamic polarization (PDP)	Easy to prepare samples [11]	Copious HE produces ohmic potential drops that are difficult to compensate for [16]
	The effect of chloride concentration on cathodic reaction can be provided [12]	Corrosion caused by PDP may alter surface and results during anodic scan [11]
	Determine instantaneous corrosion rate	Tafel fitting is too simplistic to account for several processes occurring at the electrode [17]
	Reproducible method for determination of corrosion rate	Reveal little about individual protection layers
	Shows the difference of *E*_corr_ and *i*_corr_ of alloy with different phases [12]	Investigator variation/error can cause large differences in determined corrosion current density [12]

Electrochemical impedance Spectroscopy (EIS)	Easy to prepare samples [11]	Low-frequency measurement unsuitable for rapid-corroding samples [11]
	Can be monitored continuously in real time	Difficult to choose a suitable equivalent circuit
	Samples without need to be repolished after a period of time [6]	

(Hydrogen evolution); *E*_corr_ (corrosion potential); *i*_corr_ (corrosion current density).

The article "Cross-Disciplinary Application for Qualitative Magnesium Corrosion Assays" was published in 2022. Journal: Bioinorg Chem Appl.

**Table 2:** The composition of three magnesium alloys investigated in this study.

Concentration (wt.%)	Al	Zn	Mn	Si	Ca	Fe	Mg
AZ31	2.870	0.850	0.380	0.100			Bal
AZ41	4.200	1.200	0.500	0.002	0.500	0.010	Bal
AZ91	9.210	0.800	0.340	0.060			Bal

**Table 3:** The composition of Hank's balanced salt solutions (g/L).

Component	NaCl	KCl	MgSO_4_·7H_2_O	MgCl_2_·6H_2_O	Na_2_HPO_4_·2H_2_O	KH_2_PO_4_	CaCl_2_	NaHCO_3_	Glucose
Content (g/L)	8.0	0.40	0.10	0.10	0.06	0.06	0.14	0.35	1.00

**Table 4:** Mass loss percentages of sample AZ31, AZ41, and AZ91.

Sample	AZ31	AZ41	AZ91
ML/%	0.22	0.52	0.10

## Data Availability

The data used to support findings of this study are included within the article..
